RETRACTED

# MiR-34a inhibitor protects mesenchymal stem cells from hyperglycaemic injury through the activation of the SIRT1/FoxO3a autophagy pathway

**DOI:** 10.1186/s13287-021-02183-2

**Published:** 2021-02-05

**Authors:** Fengyun Zhang, Fei Gao, Kun Wang, Xiaohong Liu, Zhuoqi Zhang

**Affiliations:** 1 Department of Cardiology, the Affiliated Hospital of Xuzhou Medical University, 99 West Huaihai Road, Xuzhou, 221000 People’s Republic of China; 2 Department of Cardiology, Institute of Cardiovascular Research, Affiliated Hospital of Xuzhou Medical University, Xuzhou, People’s Republic of China; 3 Department of Cardiology, First People’s Hospital of Suqian, Suqian, People’s Republic of China

**Keywords:** Microrna-34a, Mesenchymal stem cells, Hyperglycaemia, Senescence, Autophagy

## Abstract

**Background:**

Mesenchymal stem cells (MSCs) are favourable treatments for ischaemic diseases; however, MSCs from diabetic patients are not useful for this purpose. Recent studies have shown that the expression of miR-34a is significantly increased in patients with hyperglycaemia; the precise role of miR-34a in MSCs in diabetes needs to be clarified.

**Objective:**

The aim of this study is to determine the precise role of miR-34a in MSCs exposed to hyperglycaemia and in recovery heart function after myocardial infarction (MI) in diabetes mellitus (DM) rats.

**Methods:**

DM rat models were established by high-fat diet combined with streptozotocin (STZ) injection. MSCs were isolated from the bone marrow of donor rats. Chronic culture of MSCs under high glucose was used to mimic the DM micro-environment. The role of miR-34a in regulating cell viability, senescence and paracrine effects were investigated using a cell counting kit-8 (CCK-8) assay, senescence-associated β-galactosidase (SA-β-gal) staining and vascular endothelial growth factor (VEGF) and basic fibroblast growth factor (bFGF) ELISA, respectively. The expression of autophagy- and senescence-associated proteins in MSCs and silent information regulator 1 (SIRT1) and forkhead box class O 3a (FoxO3a) were analysed by western blotting. Autophagic bodies were analysed by transmission electron microscopy (TEM). The MI model was established by left anterior descending coronary artery (LAD) ligation, and then, the rats were transplanted with differentially treated MSCs intramuscularly at sites around the border zone of the infarcted heart. Thereafter, cardiac function in rats in each group was detected via cardiac ultrasonography at 1 week and 3 weeks after surgery. The infarct size was determined through a 2,3,5-triphenyltetrazolium chloride (TTC) staining assay, while myocardial fibrosis was assessed by Masson staining.

RETRACTED

**Results:**

The results of the current study showed that miR-34a was significantly increased under chronic hyperglycaemia exposure. Overexpression of miR-34a was significantly associated with impaired cell viability, exacerbated senescence and disrupted cell paracrine capacity. Moreover, we found that the mechanism underlying miR-34a-mediated deterioration of MSCs exposed to high glucose involved the activation of the SIRT1/FoxO3a autophagy pathway. Further analysis showed that miR-34a inhibitor-treated MSC transplantation could improve cardiac function and decrease the scar area in DM rats.

**Conclusions:**

Our study demonstrates for the first time that miR-34a mediates the deterioration of MSCs’ functions under hyperglycaemia. The underlying mechanism may involve the SIRT1/FoxO3a autophagy signalling pathway. Thus, inhibition of miR-34a might have important therapeutic implications in MSC-based therapies for myocardial infarction in DM patients.

## Background

Type 2 diabetes mellitus (DM) is a whole-body disease, and its complication cardiovascular diseases (CVDs) are the major causes of mortality in patients with DM. Diabetes develop a 2–5-fold higher risk of heart failure compared with those without [1]. Although the treatment has improved, still many DM patients die from acute myocardial infarction (MI) or suffer from follow-up heart failure, which suggests that some vital pathophysiological mechanisms have been neglected.

With the development of cell therapy research, stem cell-based cell therapy is an effective intervention for myocardial infarction. The transplantation of mesenchymal stromal cell (MSCs) plays a vital role in paracrine functions and contributes to cardiac repair through mechanisms involving cytoprotection, neovascularization and inhibition of apoptosis, all of which minimize ischaemic reperfusion injury and reduce the incidence of cardiac death and recurrent myocardial infarction [2, 3]. Yet problems of ethical, teratoma formation and immunological rejection limit the application of stem cells [4]. Among the different sources of stem cells, autologous MSCs’ treatments have shown feasibility, safety and strong indications for clinical efficacy. However, autologous MSCs from DM patient or db/db mice do not ameliorate disease symptoms compared to those from healthy individuals [5, 6]. Therefore, strategies to improve the function of MSCs in diabetic patients will become a hot topic.

MicroRNAs (miRNAs), a class of ~ 21–23 nucleotide-long noncoding RNAs, are critical repressors of gene expression through binding to the 3′-untranslated region (UTR) of target mRNAs [7]. MiRNAs have been reported to be involved in mediating multiple biological processes in stem cells, including cell division, differentiation and survival [8]. Recent studies have shown that the expression of miR-34a was significantly increased in patients with hyperglycaemia [9]. MiR-34a mediates the inhibitory effect of metformin on pancreatic tumours [10], and overexpression of miR-34a exacerbates endothelial cells’ dysfunction and decreases angiogenesis under high glucose conditions [11]. Clinical studies have shown that compared to that of control patients, miR-34a was significantly elevated in the serum of patients with myocardial infarction and diabetes mellitus, suggesting that miR-34a may be involved in the occurrence and progression of myocardial infarction and diabetes mellitus.

RETRACTED

With the development of functional studies, the maladjustment of energy metabolism in stem cells under high glucose stress leads to impaired stem cell functions and weakened abilities to repair myocardial infarction. Related studies have shown that autophagy is an important mechanism for regulating homeostasis and energy metabolism in patients with hyperglycaemia. Recently, autophagy activation was observed in a fructose-induced mouse model of ischaemia-reperfusion injury, which was associated with increased myocardial peroxidation products, fibrosis and cell death [12]. Increasing evidence had revealed that autophagy dysfunction is involved in cell death in diabetic mice. Some studies showed that autophagy could promote cell survival under hyperglycaemic conditions, while the opposite result was observed in the hearts of DM mice administered isometric corn oil by gavage [13]. These variable results prompted us to explore the precise role of autophagy in diabetic hearts.

The initiation and stability of autophagy are very complex and can be controlled by many factors. FoxO3a is an important autophagy factor. FoxO3a can be activated by AMPK, and activated FoxO3a can induce the expression of the autophagy-related proteins LC3b-II and Beclin1 and promote the expression of autophagic proteins at the site of autophagy initiation [14]. FoxO3a can also be activated by SIRT1/SIRT3, thereby activating its downstream factor PINK1, which can strongly activate PARKIN, causing mitochondrial division and activating mitochondrial autophagy, thus playing a cardioprotective role [15]. Activation of autophagy by the FoxO transcription factor may be an important way to reduce the myocardial infarction area, slow the negative remodelling of the left ventricular myocardium, promote the survival of cardiomyocytes and maintain left ventricular function [16].

The present study aimed to explore the dynamic relationship between functional changes of MSCs, autophagy and miR-34a under high glucose conditions. We hypothesized that miR-34a influenced the energy metabolism of stem cells under hyperglycaemia by regulating autophagy, thereby affecting stem cell survival, secretion and senescence, which affected the efficacy of stem cell therapy in diabetic myocardial infarction.

RETRACTED

## Materials and methods

### Reagents

Penicillin, streptomycin and HRP-conjugated goat anti-rabbit IgG (H+L) were obtained from Zhongshan Golden Bridge Biotechnology (Beijing, China), the senescent cell histochemical staining kit was obtained from Beyotime Institute of Biotechnology (Haimen, China), and the cell counting kit-8 (CCK-8) assay was obtained from Tongren Institute of Chemistry (Japan). VEGF and bFGF enzyme-linked immunosorbent assay (ELISA) kits were purchased from Wuhan Yunkelong Technology Co., Ltd. (SEA143Ra and SEA551Ra, Hubei, China). SIRT1 and FoxO3a were both from Cell Signaling Technology (#9475 and #2497, Danvers, MA, USA), LC3 was from Abcam (ab63817, Cambridge, MA, USA), Beclin1 was from Affinity Biosciences (AF5128, OH, USA) and p21 and p16 were obtained from Hua Biotechnology Co., Ltd., (ER1914-57 and ET1602-9, Zhejiang, China).

### Experimental diabetes model

All animals were housed in an accredited facility with appropriate temperature and humidity. The rats were fed standard chow. The experimental protocols were approved by Xuzhou Medical University. To establish the DM animal model, the rats were fed with high-fat diet for 8 weeks, intraperitoneally injected with streptozotocin (STZ) (25 mg/kg/d in 0.1 mM sodium citrate buffer; Sigma, St. Louis, MO, USA) and following high-fat diet for 4 weeks. Blood samples were then collected to determine the blood glucose (BG) levels using an automatic BG monitor (Lifescan Inc., Milpitas, CA, USA). Animals with fasting glycaemia levels higher than 300 mg/dl and presenting signs of polydipsia and polyuria were considered diabetic and were selected for subsequent study [17].

### Cell culture and treatments

MSCs were isolated from the bone marrow of Sprague-Dawley (SD) rats (weighing 60–80 g), as previously described. Briefly, the femurs and tibias were removed from the SD rats, and the bone marrow was washed out using 10 ml of Dulbecco’s modified Eagle’s medium/normal glucose (DMEM/L; HyClone, Waltham, MA, USA) supplemented with 1% penicillin/streptomycin (Beyotime Institute of Biotechnology, Haimen, China). The cells were centrifuged at 300×*g* for 5 min. The resulting cell pellets were resuspended in 6 ml of DMEM/L supplemented with 10% foetal bovine serum (HyClone) and 1% penicillin/streptomycin and plated in a 25-cm^2^ plastic flask at 37 °C in a humidified atmosphere containing 5% CO_2_ to allow the MSCs to adhere. After culturing the cells for 3 days, the medium was changed, and the nonadherent cells were removed. The medium was replaced every 2 days. Upon reaching 80–90% confluence, the adherent cells were detached from the dishes using 0.25% trypsin (Beyotime Institute of Biotechnology) and expanded at a dilution of 1:2 or 1:3. MSCs were characterized by flow cytometric analysis for the expression of the typical markers, CD90, CD29 and CD44 (All from BD Biosciences, Franklin Lakes, NJ, USA), and the absence of the haematopoietic markers CD45 (eBioscience, San Diego, CA, USA) and CD34 (Santa Cruz Biotechnology, Inc., Dallas, TX, USA), as previously reported [18]. MSCs from DM rat were culture under high glucose medium (25 M glucose), while MSCs from normal rat were culture under normal glucose medium (5.5 M glucose). MSCs at passage 3 were used in the experiment. For the other MSCs used in our following study, they were obtained from normal rats; for normal glucose group, the cells were cultured with 5.5 M glucose, while the high glucose group was cultured with 25 M glucose. Cells were cultured for as long as 28 days.

RETRACTED

### Cell transfection

Before transfection, MSCs were replayed into six-well plates at a density of 2 × 10^5^ cells/well and incubated overnight. For over-expression or inhibition of miR-34a, cells were transfected with 20 nM of miR-34a mimic or miR-34a inhibitor (both from GenePharma Co., Ltd., Shanghai, China), respectively. For SIRT1 inhibition, 100 nM Akt siRNA (GenePharma Co., Ltd., Shanghai, China) was transfected into cells. All miRNAs and siRNA were transfected into MSCs using a commercial transfection reagent (X-treme siRNA transfection reagent; Roche Applied Science, Penzberg, Germany) according to the manufacturer’s protocol. Forty-eight or 72 h after transfection, the cells were harvested for further analysis.

### Senescence-associated β-galactosidase staining

MSCs’ senescence was determined by in situ staining for senescence-associated β-galactosidase (SA-β-gal) using a senescent cell histochemical staining kit (Beyotime Institute of Biotechnology, Haimen, China). Briefly, after treatment, MSCs were first fixed for 30 min at room temperature in fixation buffer. The cells were washed with PBS and incubated with β-galactosidase staining solution for 16 h at 37 °C without CO_2_. The reaction was stopped by the addition of PBS. Statistical analysis was performed by counting 500 cells for each sample.

### Cell proliferation assay

Cell proliferation was assessed with the CCK-8 assay (Tongren Institute of Chemistry, Japan). For the CCK-8 assay, cells were plated onto 96-well plates (3 × 10^3^ cells/well). Assays were performed from 1 to 4 days after plating with the addition of 100 μl of fresh medium and 10 μl of CCK-8 solution for another 2 h at 37 °C. The optical density (OD) at 450 nm was measured. The assay was repeated three times.

RETRACTED

### Cytokine measurement via ELISA

Using 500 μl of supernatant containing 5 × 10^5^ cells, the VEGF and bFGF concentrations were assessed by a standard sandwich ELISA (Wuhan Yunkelong Technology Co., Ltd., Hubei, China) according to the manufacturer’s instructions. Briefly, 100 μl supernatant were transferred to the plates for 1 h at 37 °C. After washing 3 times, 100 μl reacting agent was added and was incubated for 30 min at 37 °C. After washing 5 times, the reaction was stopped by adding 90 μl chromogenic agent. The VEGF and bFGF concentrations are expressed in nanograms per millilitre and were calculated from calibration curves constructed from serial dilutions of human recombinant standards. The sensitivity of the VEGF and bFGF assays was 2 pg/ml.

### Western blotting

After the designated treatments, the cells were lysed in RIPA buffer. The protein concentration was determined with a bicinchoninic acid (BCA) kit (Beyotime, Haiman, China) according to the manufacturer’s instructions. For western blot analysis, 50–80 μg of denatured protein was separated on SDS-PAGE gels and transferred onto PVDF membranes. The membranes were blocked with 5% skim milk in TBS containing 0.5% Tween 20 (TBST) for 1 h at room temperature (RT) on a shaking table. The membranes were then incubated overnight at 4 °C with primary antibodies diluted in TBST. The membranes were subjected to three 10-min washes with TBST (TBS containing 0.5% Tween 20) and then reprobed with HRP-conjugated secondary antibodies at RT for 1 h. The membranes were then washed three times with TBST as described previously and visualized with an ECL detection system and Beyo ECL Plus reagent (Beyotime, Haimen, China), and the images were analysed using Image Lab software (version 4.1, Bio-Rad). The following antibody dilutions were used: antibodies against p21 (1:1000), p16 (308) (1:1000), SIRT1 (473) (1:1000), FoxO3a (1:1000), LC3 (1:750) and Beclin1(1:1000), and HRP-conjugated secondary rabbit antibodies (1:5000).

### Transmission electron microscopy (TEM)

MSCs with different treatment were fixed for 4 h at 4 °C in 4% glutaraldehyde (v/v) buffer, washed with 0.01 mol/L phosphate buffer solution (PBS, pH 7.0), fixed again for 2 h at 4 °C in aqueous 1% (w/v) osmium tetroxide and then embedded in Epon. Observation and photography were carried out by an electron microscope (JEM-2000EX TEM, JEOL, Tokyo, Japan).

### MI model and MSC transplantation

To induce an acute MI model, the left anterior descending coronary artery (LAD) was ligated as previously described [19]. After LAD ligation (besides the sham group), the rats randomly received one of the following treatments: (a) sham, (b) MI, (c) 3 × 10^5^ MSCs (NG), (d) 3 × 10^5^ MSCs (HG) and (e) 3 × 10^5^ MSCs (HG +miR-34a I). The group of rats that underwent thoracotomy without LAD ligation served as the sham group. All MSCs were suspended in 100 μl of PBS and injected intramuscularly at four sites around the border zone of the infarcted heart. Cardiac function in each rat was assessed by transthoracic echocardiography (Ultramark 9; Soma Technology) at baseline (before MI), and at 1 week or 3 weeks following MI. Left ventricle ejection fraction (LVEF) and left ventricular fraction shortening (LVFS) were calculated as previously described [19].

RETRACTED

### Masson’s staining

After echocardiography assessment at 3 weeks post-MI, all rats were sacrificed, and the heart tissues were harvested, embedded and sectioned. The infarction sizes of the rat hearts, as evidenced by fibrosis, were examined by a Masson’s staining kit according to the manufacturer’s protocol (HT15, Sigma). The percent infarct size was calculated as the ratio of the fibrosis area to the total LV area × 100%.

### TTC staining

2,3,5-Triphenyltetrazolium chloride (TTC) staining was performed after the heart was removed, rinsed and weighed. Next, the heart was frozen at − 20 °C for 20 min and cut into 5 sections (approximately 1–2 mm in thickness). Thereafter, the sections were subjected to a water bath containing 1% TTC phosphate buffer (pH 7.4) at 37 °C for 15 min (protected from the light and shaken) and fixed with 10% formalin. Finally, a fluorescence microscope was utilized for to capture photographs.

### Data analysis and statistics

The data are expressed as the means ± SD of at least three independent experiments. When only two value sets were compared, the statistical analysis was performed with Student’s *t* tests. The significance of differences between three or more experimental groups was determined by one-way analysis of variance. Values of *P* < 0.05, *P* < 0.01 and *P* < 0.001 were considered statistically significant, and these values are indicated by *, **, or ***, respectively.

## Results

### Hyperglycaemia damages the proliferation and paracrine abilities of MSCs

We first evaluated the effects of hyperglycaemia on MSCs. To mimic the DM micro-environment, we isolated and cultured MSCs from normal rats with high glucose for 28 days. We compared the self-renewal potential and senescence of MSCs cultured with normal and high glucose using CCK-8 assays and SA β-gal staining respectively, as well as the functional difference between MSCs from normal and DM rats.

RETRACTED

As shown in Fig. 1a and b, MSCs obtained from DM rats and high glucose-cultured MSCs exhibited decreased viability (0.51 ± 0.03 (DM group) vs.0.69 ± 0.06 (Ctrl group), *P* < 0.01, 0.49 ± 0.03 (HG group) vs.0.81 ± 0.04 (NG group), *P* < 0.01) and increased senescence (246.67 ± 20.82 (DM group) vs.100.00 ± 20.00 (Ctrl group), *P* < 0.001, 216.61 ± 20.82 (HG group) vs. 83.33 ± 20.81 (NG group), *P* < 0.001). Secretion of cytokines and growth factors to promote neovascularization is one of the major mechanisms underlying MSC-based therapy for cardiac repair after myocardial infarction [20]. In our study, we measured the level of cytokine release and found that high glucose reduced the production of VEGF (23.59 ± 3.11 (HG group) vs. 40.28 ± 8.77 (NG group), *P* < 0.05) and bFGF (30.11 ± 4.78 (HG group) vs. 59.33 ± 5.67 (NG group), *P* < 0.001) (Fig. 1c).

**Fig. 1:** Hyperglycaemia damaged the proliferation and paracrine ability of MSCs. MSCs were obtained from control or DM rats. Other MSCs were from normal rats and cultured with normal or high glucose medium for 28 days. **a** Cell viability was determined by CCK8 assay. **b** Cellular senescence was analysed by SA-β-gal staining. **c** Expression of VEGF and bFGF were measured by ELISA. **d** QRT-PCR analysis was applied to detect the expression of miR-34a. Each column represents mean ± SD from three independent experiments. *P < 0.05

These results showed that during high glucose culture, MSCs became senescent, had poor proliferation and produced fewer proangiogenic factors, which was similar to the characteristics of MSCs obtained from DM rats. In addition, to determine whether miR-34a mediates hyperglycaemic injury in MSCs, we performed qRT-PCR to measure miR-34a expression in MSCs from normal rats and DM rats and in NG- and HG-conditions (Table 1). As shown in Fig. 1d, there was a dramatic increase in the expression of miR-34a in the DM (2.60 ± 0.50 (DM group) vs.1.00 ± 0.10 (Ctrl group), *P* < 0.05) and high glucose groups (4.61 ± 0.66 (HG group) vs.1.00 ± 0.11(NG group), *P* < 0.05), suggesting a potential relationship between miR-34a and high glucose-induced damage existed.

**Table 1:** Primers for qRT-PCR and oligonucleotide

Name		Sequence
**qPCR**		
miR-34a		5′-UGGCAGUGUCUUAGCUGGUUGUU-3′
U6	F	5′-CCTGCTTCGGCAGCACA-3′
	R	5′-AACGCTTCACGAATTTGCGT-3′
	F	5′- CCCAGCACAATGAAGATCAAGATCAT-3′
	R	5′- ATCTGCTGGAAGGTGTACAGCGA-3′
**Oligonucleotide**		
miR-34a mimic		UGGCAGUGUCUUAGCUGGUUGUU CAACCAGCUAAGACACUGCCAUU
Negative Control (NC) mimic		UUCUCCGAACGUGUCACGUTT ACGUGACACGUUCGGAGAATT
miR-34a inhibitor		UGGCAGUGUCUUAGCUGGUUGUU
NC inhibitor		CAGUACUUUUGUGUAGUACAA
siRNA-SIRT1		GCACCGAUCCUCGAACAAUTT AUUGUUCGAGGAUCGGUGCTT
siRNA-NT		UUCUCCGAACGUGUCACGUTT ACGUGACACGUUCGGAGAATT

RETRACTED

### MiR-34a mediates MSCs’ dysfunction under hyperglycaemia conditions

To further analyse the relationship between miR-34a and hyperglycaemia, MSCs were transplanted with miR-34a mimic or inhibitor respectively. We first performed qRT-PCR to measure the transfection efficiency of miR-34a. As shown in Fig. 2a, when the miR-34a mimic was transfected into MSCs, the expression of miR-34a was almost 8 times higher than that in the control group (8.03 ± 0.64 (HG+miR-34a M group) vs.1.00 ± 0.10 (NG group), *P* < 0.05), but when the miR-34a inhibitor was transfected into MSCs, a significant reduction in the miR-34a level was observed (1.57 ± 0.38 (HG+miR-34a I group) vs.4.43 ± 0.42 (HG group), *P* < 0.05). Then, we performed the CCK-8 assay to examine the connection between miR-34a and cell viability under hyperglycaemia. As shown in Fig. 2b, the miR-34a mimic exacerbated the high glucose-induced damage to cell viability (0.52 ± 0.03 (HG+miR-34a M group) vs. 0.69 ± 0.06 (HG group), *P* < 0.05), while the miR-34a inhibitor alleviated high glucose-induced growth restriction (0.79 ± 0.08 (HG + miR-34a I group) vs. 0.69 ± 0.06 (HG group), *P* < 0.05).

**Fig. 2:** MiR-34a mediates MSC dysfunction under hyperglycaemic conditions. MSCs were cultured with normal or high glucose medium for 28 days with or without transfection with miR-34a mimic, NC or miR-34a inhibitor for 48 h, respectively. **a** QRT-PCR analysis was applied to detect the expression of miR-34a. **b** Cell viability was determined by CCK8 assay. **c** Expression of VEGF and bFGF were measured by ELISA. **d** Cellular senescence was analysed by SA-β-gal staining. **e** The senescence related protein of p21and p16 were determined by western blot. Each column represents mean ± SD from three independent experiments. *P < 0.05 vs. NG group. ^#^*P* < 0.05 vs. HG group

In addition, ELISA was performed to determine whether the paracrine ability of MSCs exposed to hyperglycaemia could be regulated by miR-34a. The results showed that high glucose affected the paracrine abilities and miR-34a mimic exacerbated the damage (VEGF: 21.00 ± 4.78 (HG + miR-34a M group) vs.34.14 ± 3.11(HG group), *P* < 0.05; bFGF: 19.05 ± 5.10 (HG + miR-34a M group) vs.33.11 ± 4.48 (HG group), *P* < 0.05), while the miR-34a inhibitor reversed this injury (Fig. 2c). To investigate the role of miR-34a in MSCs senescence, SA-β-gal staining and WB were performed. Compared with miR-control treatment, miR-34a mimic treatment greatly enhanced the level of SA-β-gal activity (370.33 ± 60.25 (HG+miR-34a M group) vs.199.66 ± 10.51(HG+NC group), *P* < 0.001, Fig. 2d) and the protein expression levels of p21 and p16 (p21:3.20 ± 0.10 (HG+miR-34a M group) vs.1.00 ± 0.15(HG + NC group), *P* < 0.001, p16: 4.23 ± 0.25 (HG+miR-34a M group) vs. 1.00 ± 0.18 (HG + NC group), *P* < 0.001, Fig. 2e). On the other hand, miR-34a inhibitor treatment led to an obvious increase in cell viability and decrease in the level of SA-β-gal activity (Fig. 2d) and the protein expression levels of p21 and p16 (Fig. 2e) in MSCs. Collectively, these findings suggested that the miR-34a mimic exacerbated high glucose-induced damage, while the miR-34a inhibitor protected against hyperglycaemic injury.

RETRACTED

### MiR-34a influences the expression of autophagy factors under hyperglycaemic conditions

Increasing evidence has revealed that autophagy dysfunction is involved in cell death in diabetic mice. As shown in Fig. 3a, autophagy was induced in high glucose-cultured MSCs, as evidenced by increased expression levels of Beclin-1 and LC3II/LC3I. The miR-34a mimic promoted the expression of autophagy-related proteins, as shown by western blotting (Beclin-1: 3.41 ± 0.15 (HG+miR-34a M group) vs. 2.33 ± 0.18 (HG group), *P* < 0.05; LC3: 3.55 ± 0.13 (HG+miR-34a M group) vs.1.93 ± 0.19 (HG group), *P* < 0.05, Fig. 3a), and autophagic corpuscle expression, as shown by TEM (Fig. 3c), while the miR-34a inhibitor ameliorated Beclin-1 and LC3II/LC3I expression compared with that of the control group (Beclin-1: 1.40 ± 0.14 (HG+miR-34a I group) vs.1.91 ± 0.12 (HG+NC group), *P* < 0.05; LC3:1.22 ± 0.12 (HG+miR-34a I group) vs.2.10 ± 0.15 (HG+NC group), *P* < 0.05, Fig. 3a). Collectively, these observations suggested that hyperglycaemia-induced autophagy and miR-34a mimic exacerbated this effect, while the miR-34a inhibitor decreased autophagic protein expression, which suggested that miR-34a promoted the negative effect of hyperglycaemia by regulating autophagy.

**Fig. 3:** MiR-34a influences the expression of autophagy factors under hyperglycaemic conditions. MSCs were cultured with normal or high glucose medium for 28 days with or without transfection with miR-34a mimic, NC or miR-34a inhibitor for 48 h, respectively. **a**, **b** The protein level of SIRT1 and FoxO3a, and autophagy-related protein LC3 and Beclin1 were determined by western blot. **c** Autophagic corpuscle was detected by TEM. Data are presented as mean ± SD of three separate experiments. *P < 0.05 vs. NG group. ^#^*P* < 0.05 vs. HG group

FoxO3a was reported to regulate autophagy. Our previous studies showed that the SIRT1-FoxO3a signalling pathway played a critical role in regulating apoptosis and senescence in MSCs, and we proved that SIRT1 could be negatively regulated by miR-34a expression [21]. In our study, we further examined the role of miR-34a and SIRT1/FoxO3a under hyperglycaemia conditions. The results showed that the miR-34a mimic could inhibit the expression of SIRT1 and promote the expression of FoxO3a (SIRT1: 0.18 ± 0.10 (HG+miR-34a M group) vs. 0.50 ± 0.15 (HG group), *P* < 0.05; FoxO3a: 3.97 ± 0.12 (HG+miR-34a M group) vs. 2.41 ± 0.11 (HG group), *P* < 0.05). However, whether SIRT1/FoxO3a mediates the effect of miR-34a on autophagy requires further study.

RETRACTED

### MiR-34a induces MSCs’ dysfunction under hyperglycaemia conditions by regulating SIRT1-FoxO3a autophagy dynamics

To further determine the relationship between autophagy and SIRT1-FoxO3a and the effect on cell function after exposure to hyperglycaemia, a SIRT1 inhibitor was used. As shown in Fig. 4a, treatment with siRNA-SIRT1 partially reversed the downregulation of Beclin1 and LC3II/LC3I by the miR-34a inhibitor (Belin1: 2.12 ± 0.12 (HG+miR-34a I+siRNA-SIRT1 group) vs. 1.20 ± 0.15 (HG+miR-34a I group), *P* < 0.05; LC3: 1.26 ± 0.11 (HG+miR-34a I+siRNA-SIRT1 group) vs.0.89 ± 0.13 (HG+miR-34a I group), *P* < 0.05). The SIRT1- inhibitor aggravated hyperglycaemia-induced senescence compared with miR-34a inhibitor group, as evidenced by the elevated protein expression of p21 (1.73 ± 0.22 (HG+miR-34a I+siRNA-SIRT1 group) vs.0.88 ± 0.18 (HG+miR-34a I group), *P* < 0.05) and p16 (2.11 ± 0.18 (HG+miR-34a I+siRNA-SIRT1 group) vs.1.40 ± 0.20 (HG+miR-34a I group), *P* < 0.05) and SA-β-gal activity (206.33 ± 15.82 (HG+miR-34a I+siRNA-SIRT1 group) vs.120.11 ± 10.21 (HG+miR-34a I group), *P* < 0.05). Moreover, paracrine functions were also damaged by the SIRT1 inhibitor compared with miR-34a inhibitor group (VEGF: 24.01 ± 5.12 (HG+miR-34a I+siRNA-SIRT1 group) vs. 33.18 ± 4.55 (HG+miR-34a I group), *P* < 0.05; bFGF: 26.12 ± 4.78 (HG+miR-34a I+siRNA-SIRT1 group) vs. 40.13 ± 6.25 (HG+miR-34a I group), *P* < 0.05). Overall, miR-34a regulated MSCs’ functions under hyperglycaemic conditions by targeting the SIRT1/FoxO3a autophagy signalling pathway.

**Fig. 4:** MiR-34a induces cellular dysfunction under hyperglycaemia of MSCs by regulating SIRT1-FoxO3a autophagy dynamics. MSCs were cultured with normal or high glucose medium for 28 days with or without transfection with miR-34a inhibitor or siRNA-SIRT1 for 48 h, respectively. **a** The protein expression were determined by western blot. **b** Cellular senescence was analysed by SA-β-gal staining. **c** Expression of VEGF and bFGF were measured by ELISA. Each column represents mean ± SD from three independent experiments. *P < 0.05 vs. NG, ^#^*P* < 0.05 vs. miR-34a I group

RETRACTED

### Transplantation of anti-miR-34a-MSCs improves cardiac function following infarction in diabetic rats

To examine whether the inhibition of miR-34a can improve the therapeutic effects of MSCs, we transplanted anti-miR-34a-MSCs into infarcted rat’s heart. For DM rat model, the blood glucose maintained high level compared with the normal group (Fig. 5a). MI models were successfully established in 34 rats based on the results of ECG (Fig. 5b). The 34 rats were randomly divided into five groups (6 in sham group, 7 in MI group, 7 in NG MSCs group, 7 in HG MSCs group, and 7 in miR-34a inhibitor MSCs group) respectively. The heart functions of rats in the different groups were measured by echocardiography at baseline (before MI) and 1 week and 3 weeks post-MI. At 1 week and 3 weeks post-MI, the LVEF was enhanced in MSC-transplanted groups compared with the MI group (Fig. 5b). But for the LVFS, the HG MSCs group showed little effect in elevating the heart function both in 1 week and 3 weeks, indicating the HG MSCs were limited in the ability of recovering heart function after MI. The LVEF was significantly reduced in the HG MSCs group compared with the NG MSCs group (1w: 58.23 ± 1.66 (MI+HG group) vs.68.67 ± 2.97 (MI + NG group), *P* < 0.05; 3w: 57.23 ± 3.22 (MI+HG group) vs.67.87 ± 2.47 (MI+NG group), *P* < 0.05), but this effect was partially restored in the anti-miR-34a-MSCs HG group (1w:68.70 ± 1.66 (MI+HG+miR-34a I group) vs. 58.23 ± 1.66 (MI+HG group), *P* < 0.001; 3w: 67.30 ± 1.84 (MI+HG+miR-34a I group) vs.57.23 ± 3.22 (MI+HG group), *P* < 0.05), indicating that anti-miR-34a-HG MSCs were superior to HG MSCs group in improving heart function following MI (Fig. 5b). Similarly, the infarct size, as determined by Masson’s trichrome staining, was higher in the HG MSCs group than in the NG MSCs group, while anti-miR-34a-MSCs showed improved recovery after myocardial infarction compared with the HG MSCs group (0.10 ± 0.01(MI+HG+miR-34a I group) vs.0.13 ± 0.00 (MI+HG group), *P* < 0.01). The same results were determined by TTC staining. Collectively, these findings suggest that anti-miR-34a-MSCs’ transplantation enhances heart recovery in infarcted DM rat hearts, indicating miR-34a inhibitor treatment is a favourable way for MSCs treatments for ischaemic diseases of DM rat.

**Fig. 5:** Transplantation of anti-miR-34a-MSCs improves cardiac function following infarction in diabetes rats. To establish the DM animal model, the rats were fed with high-fat diet for 8 weeks, intraperitoneally injected with streptozotocin (STZ) (25 mg/kg/day) and following high-fat diet for 4 weeks. To induce an acute MI model, the left anterior descending coronary artery (LAD) was ligated. **a** Blood glucose were determined in the DM group or the normal group. **b** ECG was taken before or after the LAD ligated. **c**–**e** Representative echocardiography images were taken at the baseline and 1 week and 3 weeks after MI. **f**–**h** Representative images of Masson’s and TTC staining were taken to detect the infarction area. Each column represents mean ± SD from three independent experiments. *P < 0.05

RETRACTED

## Discussion

The current study presented several major findings. First, hyperglycaemic culture damaged the self-renewing and paracrine functions of MSCs and exacerbated MSCs’ senescence. Second, miR-34a mediated MSCs senescence and paracrine functions by regulating autophagy. Third, miR-34a regulated autophagic dynamics under hyperglycaemic conditions by targeting the SIRT1/FoxO3a signalling pathway. Finally, the inhibition of miR-34a restored MSCs function and increased heart function and reduced the infarction area in infarcted DM rats, thereby promoting the cardioprotective effects of MSCs upon high glucose.

Over the past few decades, transplantation of MSCs has shown promising results in MI recovery in animal studies and early clinical trials due to the availability of cells from numerous sources and the multilineage potential and immune privileged status of these cells. MSC infusion is reported to ameliorate cardiac fibrosis and dysfunction in diabetic cardiomyopathy rats [22]. Besides, MSCs are verified as an effective treatment in mitigating cardiac damage by promoting angiogenesis, decreasing the infiltration of immune cells and collagen deposition in diabetes [23]. Compared with the STZ group, a significant reduction of systolic blood pressure associated with improvement of cardiac contractility was seen in the STZ/MSC rats [24]. Still several problems need to be overcome for the clinical use of stem cells, main issues include allograft immunorejection and ethics. Autologous MSCs are assumed to be favourable because patient-derived cells are readily available and do not entail sustained immunosuppressive therapy, and it has been proven that compared with those of allogeneic MSCs’ transplantation, the long-term effects of autologous MSCs are better [25]. However, MSCs isolated from DM patients become dysfunctional, as shown by changes in angiogenesis/vasculogenesis, altering pro-inflammatory cytokine secretion, increasing oxidative stress markers, impairing cellular differentiation and decreasing proliferation [26]. Furthermore, compared with healthy MSCs, DM MSCs’ transplantation exhibit impaired abilities to improve cardiac function after myocardial infarction [5].

Consistent with these observations, in the current study, MSCs isolated from DM rats displayed increased levels of SA-β-gal activity and decreased proliferative and paracrine capacities. We also observed that high glucose-cultured MSCs exhibited almost the same behaviour as DM MSCs, and so in the following studies, MSCs treated with chronic exposure to high glucose for 28 days were used to mimic the behaviour of DM MSCs. However, the potential mechanisms underlying DM MSCs’ dysfunction remained unclear.

RETRACTED

Recently, a variety of miRNAs have been reported to be involved in regulating MSCs’ function during heart recovery process after myocardial infarction [5]. Among the known miRNAs, miR-34a has been implicated in cardiovascular diseases such as atherosclerosis, ischaemic cardiomyopathy and myocardial infarction. Recent studies have shown that the expression of miR-34a is significantly increased in patients with hyperglycaemia [9]. MiR-34a mediates the inhibitory effect of metformin on pancreatic tumours [10], and overexpression of miR-34a exacerbates endothelial dysfunction and decreases vasculogenesis under high glucose exposure [11]. Our previous results showed that the expression of miR-34a was significantly increased in the ischaemic/hypoxic environment (used to simulate the hypoxic and ischaemic microenvironment in myocardial infarction), the activity of MSCs with miR-34a overexpression was decreased, the apoptosis rate was significantly increased, and cell senescence was also increased in the ischaemic and hypoxic environment. However, it has not been reported whether miR-34a affected the functional changes in MSCs exposed to high glucose.

In the present study, miR-34a was markedly increased under hyperglycaemia conditions. We further found that over-expression of miR-34a in MSCs exposed to hyperglycaemia enhanced the senescent phenotype, including increased SA-β-gal activity and expression of p21 and p16. Besides, miR-34a mimic treated MSCs under hyperglycaemia also shown decreased proliferative and paracrine capacities. In contrast, inhibition of miR-34a in MSCs exposed to hyperglycaemia reduced SA-β-gal activity, increased cell proliferation and promoted the secretion of VEGF and bFGF. Transplantation of anti-miR-34a-MSCs had better effects in attenuating cardiac remodelling and restoring heart function in DM rats following infarction than transplantation of MSCs cultured in high glucose.

These findings confirmed that miR-34a accelerated MSCs’ dysfunction in hyperglycaemia and that inhibition of miR-34a restored MSCs’ abilities. The exact mechanism underlying miR-34a-mediated regulation of MSCs function, however, is still largely unknown.

Autophagy is an evolutionarily conserved mechanism by which cytoplasmic elements are degraded intracellularly. Autophagy has emerged as a major regulator of cardiac homeostasis and function. Autophagy was demonstrated to promote the paracrine secretion of VEGF in MSCs [27]. Suppressed autophagy contributed to the progression of heart failure (HF) and ageing [28]. On the other hand, autophagy activated excessively under ischaemia/reperfusion and the acute phase of pressure overload may facilitate myocardial injury [29]. The above controversial effect of autophagy can also been seen in type 2 diabetic hearts. On the one hand, suppression of autophagy could induce cell death, fibrosis and dysfunction in type 1 diabetic hearts [30]. On the other hand, promotion of autophagy expression can express more VEGF for MSCs’ treatment to better ameliorate erectile dysfunction [31]. Also, cardiomyocytes isolated from db/db mice [32] and HFD-induced obese mice exhibited blunted autophagic responses [33]. In the present study, during hyperglycaemia culture, MSCs exhibited excessive antophagy, as evidenced by over-expression of LC3 and cytolysosome. Moreover, when we inhibited the expression of miR-34a, the phenomenon was reversed. Excessive expression of autophagy was one of the most important mechanisms that was involved in miR-34a’s role on MSCs’ dysfunction under hyperglycaemia.

RETRACTED

The initiation and stabilization of autophagy was a complex process regulated by many factors in the micro-environment, of which FoxO3a was an important factor. FoxO3a was a member of the FoxO transcriptional family. FoxO3a activation induced autophagy gene expression and decreased cardiomyocyte cell size [34]. FoxO3a could also be directly targeted by miRNA-212/132, and over-expression of these miRNAs led to an impaired autophagic response upon starvation and promoted hyper-activation of pro-hypertrophic calcineurin/ NFAT signalling [35]. In response to stress or pathological conditions, FoxO3a could be phosphorylated by SIRT1 and was retained in the cytosol, thereby inhibiting its transcriptional activity [36]. Activation of SIRT-1 promoted the transcription of genes that regulated mitochondrial biogenesis to maintain energy and metabolic homeostasis [37, 38]. SIRT-1 deacetylated members of the forkhead box O (FoxO) family and affected downstream pathways controlling autophagy [39, 40]. Pharmacological stimulation of SIRT-1 attenuated hepatic ischaemic/reperfusion injury through mitochondrial recovery and enhanced autophagy [41].

The relationship between miR-34a and SIRT1 and FoxO3a had been described in our previous study that during hypoxia and serum deprivation, over-expression of miR-34a led to robust apoptosis regulated by SIRT1/FoxO3a pathway activation [21]. In the current study, we found that the expression of SIRT1 was greatly decreased in high glucose-induced MSCs compared with the normal MSCs. Furthermore, miR-34a mimic treatment greatly reduced the expression of SIRT1 and increased FoxO3a expression and promoted the expression of autophagy. Moreover, we found that siRNA-SIRT1 partially reversed the effect of miR-34a inhibitor on inhibiting excessive autophagy induced by hyperglycaemia. These results further confirmed that miR-34a induces autophagy by partially targeting SIRT1/FoxO3a signalling.

RETRACTED

The predominant mechanism of MSCs to exert a therapeutic effect on MI is paracrine. Transplanted MSC-derived endothelial cells and vascular smooth muscle cells can contribute to the new vessel formation [42]. MSCs’ paracrine factors include protein cytokines such as VEGF, hepatocyte growth factor (HGF), insulin-like growth factor (IGF), miRNAs [43] and exosomes [44]. The VEGF and bFGF have a strong proangiogenic effect, due not only to promotion of endothelial cell proliferation and migration but also to prevention of endothelial cells from apoptosis [45].

The relationship between autophagy and angiogenesis has been discussed in some aspects. Inhibiting autophagy by ATG5/7 knockdown decreased the levels of angiogenin and VEGF expression upon hypoxia exposure [46]. Other study demonstrated that increased spontaneous production of VEGF may induce angiogenesis after MI through initiating autophagy in the vascular endothelial cells [47]. In the present study, during hyperglycaemia process, we could see that the paracrine function was damaged indicating by reduced expression of VEGF and bFGF. But when the miR-34a inhibitor was used to inhibit the over-excessive of autophagy, the release of VEGF and bFGF were increased.

In vivo experiment further detected the effect of miR-34a on the stem cell therapy on DM myocardial infarction. The stem cell-mediated repair of myocardial infarction under different treatment conditions was observed in rats. The DM MI rat showed reduced LVEF, severe fibrosis and larger infarction area, which partly explained the vital issue that in clinical the diabetic myocardial infarction showed high mortality than those without [48]. MSCs cultured under normal glucose showed ability to reduce this damage; however, as is shown in Fig. 5c, MSCs cultured under high glucose medium showed little effect in recovery the heart. When the miR-34a was inhibited in the MSCs upon hyperglycaemia, the MSCs’ function was elevated and the ability to reduce the infarction area was also increased. Suggesting that miR-34a inhibitor could protect mesenchymal stem cells from hyperglycaemic injury and provided a promising role for autologous transplantation of MSCs for DM myocardial infarction patients.

RETRACTED

This project examined the effects of miR-34a on the function of MSCs upon high glucose, including proliferation, senescence and paracrine signalling and the relationship between miR-34a and the SIRT1-FoxO3a-autophagy signalling pathway. We found that miR-34a expression increased in MSCs under long-term high glucose exposure and then affected the energy metabolism pathway of autophagy. MiR-34a inhibitor alleviated the damage of hyperglycaemia on MSCs both in vitro and in vivo studies. Transplantation of anti-miR-34a-MSCs could elevate the LVEF function and reduce the fibrosis and infarction area, which promoted heart recovery in myocardial infarction in diabetes rats. The anti-miR-34a-MSCs’ therapy maybe have wide clinical applications for patients with myocardial infarction and diabetes.

### Conclusion

This study demonstrates that inhibition of miR-34a, which occurs partially via the SIRT1/FoxO3a autophagy-signalling pathway, restores damaged MSCs exposed to hyperglycaemia and provides a possible target to enhance the cardioprotection of MSCs in the DM heart following infarction.

## Data Availability

The datasets used and/or analysed during the current study are available from the corresponding author on reasonable request.

## Abbreviations

MSCs: Mesenchymal stem cells
CCK8: Cell counting kit-8
STZ: Streptozotocin
DM: Diabetes mellitus
SA-β-gal: Senescence-associated β-galactosidase
SIRT1: Silent information regulator 1
FoxO3a: Forkhead box class O 3a
VEGF: Vascular endothelial growth factor
bFGF: Basic fibroblast growth factor
TEM: Transmission electron microscopy
LAD: Left anterior descending coronary artery
TTC: 2,3,5-Triphenyltetrazolium chloride
CVDs: Cardiovascular diseases
MI: Myocardial infarction
BG: Blood glucose
SD: Sprague-Dawley
BCA: Bicinchoninic acid
LVEF: Left ventricle ejection fraction
